The article "Research on the Application of GIS Technology Combined with RBFNN-GA Algorithm in the Delineation of Geological Hazard Prone Areas" was published in 2021. Journal: Comput Intell Neurosci.

# Research on the Application of GIS Technology Combined with RBFNN-GA Algorithm in the Delineation of Geological Hazard Prone Areas

**DOI:** 10.1155/2021/2677453

**Published:** 2021-12-02

**Authors:** Tianwang Lei, Yao Lu, Chong Zhang, Jing Wang, Qi Zhou

**Affiliations:** ^1^School of Civil Engineering, Xi'an Traffic Engineering Institute, Xi'an, Shannxi 710300, China; ^2^School of Geography and Environment, Baoji College of Arts and Sciences, Baoji, Shannxi 721013, China

## Abstract

With the rapid development of the economy and society, geological disasters such as landslides, collapses, and mudslides have shown an intensifying trend, seriously endangering the safety of people's lives and property, and affecting the sustainable development of the economy and society. Aiming at the problems of merging different data layers and determining the weighting of data stacking in the statistical analysis model based on GIS technology in the evaluation of the risk of geological disasters, this study proposes a logistic regression model combined with the RBFNN-GA algorithm, that is, the determination of the occurrence of geological disasters. The fusion coefficient (CF value) with the RBFNN-GA algorithm model, and with the help of SPSS statistical analysis software, solves the problem of factor selection, heterogeneous data merging, and weighting of each data layer in the risk assessment. In the experimental stage, this study adopts the method of geological hazard certainty coefficients to carry out the sensitivity analysis of the geological hazards in the study area. Using homogeneous grid division, the spatial quantitative evaluation of the risk of geological disasters is realized, and at the same time, the results of the spatial quantitative evaluation of the risk of geological disasters are tested according to the latest landslide points in the region. The existing classification mainly depends on the acquisition of land use/cover information or the processing method of the acquired information, but the existing information acquisition will be limited by time, space, and spectral resolution. The results show that the number of landslide points per unit area in the extremely unstable zone and the unstable zone is 0.0395 points/km^2^ and 0.0251 points/km^2^, respectively, which is much higher than 0.0038 points/km^2^ in the stable zone, indicating the evaluation results and actual landslide conditions.

## 1. Introduction

According to statistics, in the past 50 years, landslides, collapses, and mudslides have caused more than 20,000 deaths, with hundreds to more than 1,000 deaths every year. Among the many natural disasters, the death toll is second only to earthquakes and floods. In particular, landslides, collapses, and mudslides that erupt in densely populated areas such as towns and mining areas often cause a disaster event that kills hundreds of people [1]. Geological disasters such as landslides, collapses, and mudslides are one of the natural disasters that cause the loss of people's lives and property [2]. In order to effectively prevent and reduce geological disasters, it is first necessary to have a more comprehensive understanding of regional geological disasters. When formulating regional geological disasters, they can be more targeted. At the same time, research on geological disaster forecasting and early warning is based on the division of geological disasters. The foundation has also become a hot issue in the field of geological disaster research [3]. There are many domestic studies on the mechanism of single geological disasters such as landslides, but the research progress on the development and distribution of regional geological disasters is relatively slow [4]. Exploring and forming a set of scientific, complete, and practical research methods for the development and distribution of regional geological disasters, and evaluating the risk of regional geological disasters, is of great practical significance for the prevention and control of regional geological disasters [5].

The article "Research on the Application of GIS Technology Combined with RBFNN-GA Algorithm in the Delineation of Geological Hazard Prone Areas" was published in 2021. Journal: Comput Intell Neurosci.

The geological hazard evaluation method adopted at the beginning has inherited the evaluation of geography in many methods, and the methods used can be summarized as follows: dominant factor method, multifactor single-factor item-by-item overlay method, geographic correlation analysis method, and theoretical derivation method [6]. After the 1980s, the degree of quantification increased, the application of mathematical knowledge in geosciences developed vertically and horizontally, and the geological hazard evaluation and zoning research gradually tended to quantify [7]. The extensive application of linear regression prediction, mathematical model analysis, gray theory, neural network, GIS, etc. is gradually introduced to further improve the degree of quantification [8]. In the study of slope geological hazards in an urban development planning project in Australia, Mai [9] integrated the risk, vulnerability, and risk assessment of slope hazards, using GIS software as the technical platform, and using two-dimensional and three-dimensional evaluation systems, respectively, for research on the danger and risk zoning of slope geological disasters in Cairns area. He et al.'s [10] probabilistic analysis and forecasting models show that these models have their own advantages but also have certain shortcomings. For example, the models established by index analysis methods, probability statistical methods, and fuzzy prediction methods are generally only suitable for specific research. At the same time, it is difficult to extract information related to the geology, mechanics, and other environmental conditions of the sliding mass. Liu [11] applied a genetic algorithm to the neural network to form the GA-ANN method to collaboratively solve optimization problems in complex engineering. This method not only uses the functions of neural network's nonlinear mapping, network reasoning, and prediction but also uses the global optimization characteristics of genetic algorithm. It can be widely used in many complex projects where the objective function is difficult to express in the form of explicit function of decision variables. Peng [12] applied the genetic algorithm to the artificial neural network model to determine the maintenance strategy of the parts and analyzed it in combination with examples. After experimental verification, the system selected the maintenance strategy and the actual value is in full compliance with the relative error between the predicted value of the maintenance cost and the actual value. Within the allowable range, the model is credible. Afan [13] applied the genetic algorithm to optimize the parameters of the controller based on the neural network structure and used the controller to control the objects with pure lag. The experiment proved that the control system optimized by the genetic algorithm has good static performance and dynamics. Performance has made a new exploration for solving this problem in the control field. The background factors include engineering rock formations, topography, geological structure, seismic intensity, human engineering activities, and atmospheric precipitation [14–16].

The article "Research on the Application of GIS Technology Combined with RBFNN-GA Algorithm in the Delineation of Geological Hazard Prone Areas" was published in 2021. Journal: Comput Intell Neurosci.

This study takes the regional geological disaster survey project of the autonomous region as the background, based on abundant actual data, deeply researches various factors affecting the occurrence of geological disasters, comprehensively analyzes the relationship between the distribution of geological disasters and various factors, and explores the determination of regional geological disasters. They should have the same or similar spectral information features and spatial information features, so the feature vectors of the pixels of the same type of features will be clustered in a unified feature space area, and different features will be due to different spectral information features or spatial information features. The method of risk has established a risk assessment system for regional geological disasters. Studies have shown that the regional layered soft phyllite intercalated with hard sandstone rock formations, a slope of 20°–40°, and an elevation range of 320–800 m above sea level are most prone to geological disasters. The key factors affecting the risk of geological disasters are elevation, rock formations, road construction, and slope. According to the calculated cell geological hazard probability value, the regional geological hazard risk is divided into 4 levels, namely, extremely unstable, unstable, basically stable, and stable.

## 2. GIS Technology Based on RBFNN-GA Algorithm in the Delineation Model Construction of Geological Hazard Prone Areas

### 2.1. GIS Technology Level Classification

Geographic information system (GIS) is a decision support system that collects, stores, manages, analyzes, and reproduces information related to geographic spatial distribution and has various characteristics of an information system [17]. The main difference between geographic information system and other information systems is that the information stored and processed by it is geocoded. Geographic location and related feature information become an important part of information retrieval.  Figure 1 shows the hierarchical topology of GIS technology.

The most important part of the geographic information system is spatial data. Spatial data can effectively express spatial location information and attribute data, while GIS spatial database is a collection of spatial data reasonably stored. The spatial database management system developed on this basis can effectively provide spatial query and analysis [18–20]:

(1) $$\begin{array}{c} p\left(x\left(1\right),x\left(2\right),\ldots ,x\left(n\right)\right)=\prod_{i=1}^{n}p\left\{x\left(n\right)|x\left(n-i+1\right)\right\}. \end{array}$$

In MapX, all the features in a layer constitute a feature set. Each graphic element is a feature object (Feature), and many methods of the layer object (Layer) return the feature set of the layer. You can search and locate geographic features such as lines, symbols, or regional characteristics [21–24]. In order to be able to use this method, there must be an index field in the MapInfo table of the search layer:

(2) $$\begin{array}{c} f\left(x\right)=x\left(i\right)+\frac{x\left(i\right)\times x\left(j\right)}{x\left(i\right)+x\left(j\right)},\\ T^{2}-\frac{1}{n}\times \overset{n}{\underset{i=1}{\sum }}{\left(p\left(i\right)-p\left(x\right)\right)}^{2}=0. \end{array}$$

The basic building blocks of MapX components are a single object and a collection. The collection includes objects, which is a combination of multiple objects. Each kind of alignment and collection is responsible for processing a certain aspect of the map. In the model structure of MapX, the Map object exists at the top, and each MapX object, attribute, and method are derived from the Map object.

(3) $$\begin{array}{c} \left\{\begin{array}{c} x\left(i,0\right)=a-x\left(j,0\right),\\ x\left(i,1\right)=b-x\left(j,1\right),\\ x\left(i,j\right)=\sqrt{\frac{x\left(j,i\right)}{a+b}.} \end{array}\right. \end{array}$$

Each attribute and method under the Map object will have an impact on the generation of the entire Map object. Each Map object is mainly defined by DataSets, Layers, and Annotations objects. Among them, Layers are mainly used to manipulate the layers of the map, DataSets are used to access spatial data tables, and Annotations are used to add text and symbols on the map:

(4) $$\begin{array}{c} S\left(x,m\right)-\frac{\left(1/2\right)\times x\left(m\right)p\left(n\right)+\left(2/3\right)\times x\left(n\right)p\left(m\right)}{p\left(m\right)+p\left(n\right)}=0,\\ I=\left\{\text{C}\left(x,y\right)\text{,}x\in \left(0,1,2,\ldots ,n\right),y\in \left(0,1,2,\ldots ,n-1\right),n\in N\right\}\text{.} \end{array}$$

The basic idea of GIS is to divide the main functional modules of GIS into several components, and each component performs different functions. Various GIS components, as well as between GIS components and other non-G1S components, can be easily integrated through visual software development tools to realize the final GIS application [25–27]:

(5) $$\begin{array}{c} L\left(x,y\right)=\sqrt{{\sum \left[C_{a}\left(x,y\right)-C_{b}\left(x,y\right)\right]}^{2}}. \end{array}$$

Each map has a data set. Through the data collection, the user's attribute data can be connected with the map spatial data. Data binding is the process of introducing external data into MapX. External data can be multiple types of databases.

(6) $$\begin{array}{c} K\left(x,y\right)=\left[\begin{array}{cc} k\left(x\right)\times \;\cos\;x & 1\\ 1 & k\left(y\right)\times \;\sin\;y \end{array}\right]. \end{array}$$

After data binding, you can browse the data on the map as primitives or create a thematic rendering map based on these data. The learning process consists of three stages. The first stage uses unsupervised methods to determine the center of the RBF; the second stage determines the width of the RBF based on the determined center of the RBF; and the third stage determines the distance between the intermediate layer and the output layer. Generally speaking, these stages are carried out separately.

The article "Research on the Application of GIS Technology Combined with RBFNN-GA Algorithm in the Delineation of Geological Hazard Prone Areas" was published in 2021. Journal: Comput Intell Neurosci.

### 2.2. The Composition of Geological Hazards

Geological disaster refers to a disaster related to geological action caused by natural factors or human engineering economic activities, which damages the ecological environment and endangers the safety of human life and property. It is in the shape of an inverted stone cone, with a loose and disorderly structure. The dangerous rock mass is a dangerous mountain mass that is cracking and deforming, and may collapse. Landslide refers to the phenomenon that the rock and soil on the slope lose the original balance condition and move downward along a certain weak surface as a whole or scattered along a certain weak surface under the influence of river erosion, groundwater activity (heavy rain), earthquake, and artificial slope cutting. The tendency of the weak structure surface is consistent with the slope direction, and the slope angle is most likely to occur when the slope angle is greater than the inclination angle of the weak surface. The material can be a loose layer, soft rock, and hard rock. A complete landslide should have a sliding surface (slide bed), landslide surface cracks and steps, trailing and lateral sliding walls, cracks, and front bulging. The influencing factors and formation conditions of geological disasters are extremely complex. They act independently, but also influence and overlap each other. According to their active forms, they are summarized as influencing factors and basic conditions; influencing factors include atmospheric rainfall, hydrogeology, neotectonic movement, and human activities; the basic conditions include topography and geomorphology conditions, stratum lithology conditions, and geological structure conditions. The spatial database of this project includes spatial databases of engineering geology and geological disasters.  Figure 2 shows the fan chart of the factors of geological hazards.

This database system is constructed in accordance with the relevant provisions. The system includes geological hazard field survey data, result data, its spatial graphic database, and database structure, and the naming of format, layer, view project file, and the structure of primitive number are all carried out in accordance with regulations. The research area has a relatively complete range of disasters. Based on the geological environmental conditions formed in the area, the degree of disaster susceptibility, the degree of harm, and the integrated social development plan, a comprehensive analysis is made. The research area is divided into key prevention and control areas, subkey prevention and control areas, and general prevention area. We adopt measures such as restoring vegetation, cutting slopes, clearing dangerous rocks, strengthening supports, monitoring and forecasting of ground collapse disaster areas, strengthening of the survey of building foundations, assessment of the risk of geological disasters in disaster areas, and dredging of debris flow disaster areas. For river courses, excavation of water-cutting ditches around mountains, construction of slope protection, valleys, blocking dams, etc., the long term should be based on biological engineering and engineering treatment. According to geological survey data, the probability of geological disasters on concave slopes in the study area is low, and the probability of geological disasters on linear and convex slopes is greater. When the slope of convex slopes in the area is more curved, the relatively concentrated stress of the slope ultimately affects the stability of the slope. Therefore, the shape of the slope directly affects the possibility of geological disasters in the study area.

The article "Research on the Application of GIS Technology Combined with RBFNN-GA Algorithm in the Delineation of Geological Hazard Prone Areas" was published in 2021. Journal: Comput Intell Neurosci.

### 2.3. RBFNN-GA Algorithm Design

The RBF neural network is a forward neural network that combines a parameterized statistical distribution model and a nonparametric linear perceptron model. The essence of the RBF neural network is the combination of unsupervised clustering method and supervised single-layer linear perceptron to realize the neural network model of nonlinear mapping. The RBF neural network is composed of 3 layers, namely, the input layer, the middle RBF layer, and the output layer. For hyperspectral images, it is difficult to get so many pixels in a limited space for certain classes, and as the dimensionality of the feature space increases, the accuracy degradation called the Hughes phenomenon also requires more training samples. Generally, the number of nodes in the input layer is equal to the dimension of the selected data in the application field, and the number of nodes in the output layer is equal to the number of categories to be classified. For a specific application, the number of nodes in the input layer and output layer is determined. Therefore, the design of the RBF network structure is mainly to determine the number of nodes in the middle RBF layer. It uses the connection strength and the nonlinear input-output relationship of neurons to realize the nonlinear mapping from the input state space to the output state space. Feedforward networks are widely used in pattern classification and feature extraction. Another mode of operation is evolutionary, in which the input is equivalent to the initial state, and the final state of network evolution is the output. This kind of network is similar to a dissipative nonlinear dynamic system.

Figure 3 shows the RBFNN-GA algorithm architecture. The state space shrinks continuously during evolution and finally shrinks to a small attracting subset, and each attracting subset has a certain attraction domain. The energy function is a basic quantity of this type of network. Using the local minima of the energy function, operations such as associative memory, information compression, and coding can be performed: only the global minima of the energy function can be used to solve combinatorial optimization problems, such as TP problems, visual matching, and problem-solving. Output layer learning is a kind of supervised learning. In supervised learning, the attributes of the pattern samples to be classified are known, and for each sample input and output, there is a corresponding guidance signal that matches its nature. Based on the network output supervision, the various objective function criteria of the signal and the actual output adjust the weights accordingly until the accuracy reaches the best requirements. The database is based on the implementation project, the standard map sheet is the spatial index, and the geological disaster professional data are classified as the first-level processing object. According to the storage form, it is divided into two parts: the graphic database and the attribute database. Respective graphic elements and associated fields of records (or unified numbers) realize the two-way dynamic connection, combined with multimedia database and graphical legend data, to lay the foundation for environmental geological survey and evaluation as the application goal. The specific operation is carried out in strict accordance with the input direction and input sequence in the technical requirements of spatial database construction and the method of distinguishing different line elements with different colors to form a comprehensive graphic line file in order to facilitate the hierarchical extraction of line files.

The article "Research on the Application of GIS Technology Combined with RBFNN-GA Algorithm in the Delineation of Geological Hazard Prone Areas" was published in 2021. Journal: Comput Intell Neurosci.

### 2.4. Delineation of Regional Features

The Permian and Triassic strata are the most widely distributed in the area. Among them, the Triassic strata are the most well developed. Carbonate rocks account for about 68% of the total thickness of the strata. Carbonatite and clastic rocks are multilayered in vertical distribution and are also called interbedded carbonate rocks. The interbedded carbonate rocks are distributed in a strip-like plane. That is to say, except for the Yanshan Movement, which is an obvious fold orogenic movement, the rest of the crustal movement is slowly ascending and descending. Therefore, the regional crust is relatively stable. In order to apply the projection transformation of GIS, we first transform the data format in the database.  Figure 4 shows a quantitative histogram of the susceptibility of geological disasters.

The grid map of the susceptibility of geological hazards is obtained through spatial analysis and superposition based on the changing trend of geological hazard points. The stability of regional landslides, avalanches, ground subsidences, and unstable slopes is divided into three categories: unstable, basically stable, and stable using expert assessment methods; for debris flows, the integral method is used, and the evaluation factor is determined to be 15 items. The integral value method is used to assess the susceptibility of debris flow geological hazards. Taking the 1 : 100,000 topographic map of the study area as the basic base map, it is divided by the raster data processing method. Taking into account the geological environment and disaster development status of an area, the standard area grid is 2 km × 2 km. The area is divided into 66 rows and 6l columns, with a total of 1,856 cells. Compared with traditional computer remote sensing classification, its classification accuracy is significantly improved, providing technical reserves and references for land use dynamic monitoring and land use management. Using the face-to-point intersection function of GIS spatial analysis, the face-to-point intersection calculation is performed between the surface file of the divided grid and the point file of various disaster points (with the attribute of proneness degree) to obtain different levels of disasters. Each cell is assigned a value based on the highest level of a type of disaster point that appears in the range. Using the method of GIS spatial analysis, the surface files of the divided grid and the point files of various geological disaster points (with the attribute of proneness degree) are calculated to obtain the partition files of different levels of various disasters. The partition files of different levels of various disasters obtained above are superimposed according to the following formula, which is the result of the scoring area. First, we superimpose the files in various unstable or high-prone areas. When there are two or more geological hazard high-prone areas overlapping, the value is 5. Second, we intersect all kinds of basically stable or medium-prone surface files with the merged unstable or high-prone surface files, subtract the common parts, and superimpose and merge according to the above formula to obtain the medium-prone layer. Third, we intersect all kinds of stable or low-prone surface files with the merged high- and medium-prone files and subtract the intersecting part, superimpose, and merge according to the above formula to get the low-prone layer. Finally, we subtract the high-, medium-, and low-prone areas from the whole picture, and the remaining areas are less prone areas. After merging, the zoning grid map of the susceptibility of the whole area can be obtained.

The article "Research on the Application of GIS Technology Combined with RBFNN-GA Algorithm in the Delineation of Geological Hazard Prone Areas" was published in 2021. Journal: Comput Intell Neurosci.

## 3. Application and Analysis of GIS Technology Based on RBFNN-GA Algorithm in the Delineation Model of Geological Hazard Prone Areas

### 3.1. RBFNN-GA Algorithm Data Extraction

The hardware requirements of this system are as follows: CPU Pentium 1.5 GHz, memory 512 M, hard disk 20 G and above running on computers, Windows 2000/XP/2003 operating system, and software platforms that mainly include ERDAS IMAGINE 8.7, MATLAB 6.5, and Visual Studio 2005. Through field surveys and referring to the current land use map, we select typical land use plots and record their latitude and longitude coordinates. We use the remote sensing image file and text file conversion tool provided by ERDAS IMAGINE to convert the established training sample area into a text file; use the text file reading function provided by MATLAB to write the band values of each land use type into the matrix; and build a network model through the newrb function. The results of the network simulation are output in the form of a matrix, and when the accuracy analysis and classification results are evaluated, the image map is used as the basic data. Therefore, the classification results in the matrix form should be converted and restored into remote sensing images. This work can be done through remote sensing.

Figure 5 shows the normalized comparison line chart of RBFNN network evaluation indicators. We integrate the normalized results of the aforementioned various evaluation index data analysis and then use all the indicator inputs by the spatial overlay and analysis function in ArcGIS to obtain the digital matrix result; in ArcGIS, the Raster Calculator distributes the index data in the study area according to the weight. After the stacking calculation, the results need to be reclassified. Using the natural discontinuity grading method in the classical tool in ArcGIS, the stacking results are divided into three levels, and the regional geological hazard risk assessment result map is obtained. The system function mainly includes the selection of training sample area and the establishment of RBFNN algorithm and simulation. According to the scores in the result map superimposed by various indicators of the region, the geological hazard risk is divided into three levels, namely, high, medium, and low, and then according to the actual situation, the repeated operation of grid or merging small redundant areas is performed. Finally, an artificially modified and integrated geological hazard risk zoning map can be obtained. The data calculated by GIS technology have been obtained by statistics of 16 villages and towns in the region. The requirement of consistency requires the establishment of a new judgment matrix through the relationships at all levels until the calculation and judgment results are reasonable. According to the principle of checking the consistency of the judgment matrix, matrix 1, matrix 2, matrix 3, and matrix 4 are calculated and tested, respectively, and the average CR < 0.1 is obtained. It is known that the constructed regional geological disaster risk assessment judgment matrix meets the consistency requirements.

The article "Research on the Application of GIS Technology Combined with RBFNN-GA Algorithm in the Delineation of Geological Hazard Prone Areas" was published in 2021. Journal: Comput Intell Neurosci.

### 3.2. Realization of GIS Delineation in Areas Prone to Geological Hazards

In this study, the neural network was set with 6 input nodes and 1 output node, and the initial value of the hidden node was 20. We used the control force to train the network parameters. The number of SGA implicit function nodes is fixed as 6, and the crossover probability is 0.7. The probability of variation is 0.05. The maximum fitness value changes during the training process as described in the text. As the core part of the geographic information system, the design quality of the database will not only affect the cost and quality of the system construction but also affect the operation, maintenance, and data update of the system. At the same time, the content and structure of the database determine the quality of the system and will have a direct impact on the integration of GIS and other application technologies. When designing the system, we fully consider the scalability and compatibility of the system. In terms of the encoding of disaster-type information, the selection of the base map coordinate system, the design of the database, and the system interface functions, as much as possible, there is room for further development to facilitate the expansion of the system. With database migration, when new modules are added, the functional structure of existing modules and the entire system will not be greatly affected.

Figure 6 shows the distribution of curvature of geological hazards in the GIS system. According to the survey of geological disasters, the probability of geological disasters on concave slopes is relatively small, while the probability of geological disasters on straight and convex slopes is greater. The more curved the slopes of convex slopes are, the more concentrated the stress on the slope is. Therefore, for the slope curvature, when the curvature of a certain area is less than 0, the possibility of geological disasters is smaller. A large number of human engineering activities have a direct or indirect impact on the formation and development of landslides, collapses, and unstable slopes in the study area. Considering that traffic construction such as roads and railways is the most representative human engineering activity in the region, it has the most impact on geological disasters. Obviously, it has the characteristics of penetration and full coverage, so the analysis of human engineering activities in this study takes the regional secondary road as the baseline and makes buffer analysis. A value close to 0 means that the prior probability is very close to the conditional probability, and the certainty of the occurrence of the event is close to the regional average. When the curvature is greater than 0, the possibility of geological disasters is high, and the greater the curvature is, the more unstable the slope is. We use the Raster Calculator in ArcGIS to do the difference to calculate the slope height index map of the study area. Finally, it can be normalized by Raster Calculator in ArcGIS.  Table 1 shows normalized processing of GIS disaster indicators.

The article "Research on the Application of GIS Technology Combined with RBFNN-GA Algorithm in the Delineation of Geological Hazard Prone Areas" was published in 2021. Journal: Comput Intell Neurosci.

The improved HANHGA-trained neural network controller and the SGA-trained neural network controller were used to control the double-stage inverted pendulum, and the simulation block diagram of the entire control system was built in Simulink using MATLAB. It can be seen that the improved HANHGA has a faster convergence speed and higher accuracy. The improved HANHGA training neural network has an error of 4.2% when it is trained for 100 generations, while the error of the SGA training neural network is only at the end of 200 generations. It reaches 1.2%, so the improved genetic algorithm has greater advantages than a simple genetic algorithm in convergence speed and in finding the global optimal solution. As a comparison between the improved HANHGA's RBFNN control method and the SGA neural network control method, it can be seen that the improved RBFNN control method can restore the inverted pendulum to a stable state faster, which proves the superiority of the improved algorithm. The data in the figure represent the control effect of the improved algorithm. It can be seen that it has a smaller overshoot and a shorter settling time, which proves the superiority of the improved algorithm.

### 3.3. Example Application and Analysis

On the ERDAS IMAGINE platform, using the Image Interpreter function provided by it, in the Utilities menu, the layer overlay module completes the overlay of each monochrome band, the data type is output as unsigned 8-bit data, and image fusion is mainly performed in the Spatial Enhancement menu. The fusion method uses a principal component (principal component analysis), and the resampling aspect is cubic convolution sampling. The key technologies for image geometric correction mainly include the selection of digital geometric correction calculation models and ground control points. For the determination of the gray value of the digital image and the resampling of the gray value of the digital image, the selection of the resampling method is particularly important. The commonly used gray value resampling methods mainly include the nearest point method, the bilinear interpolation method, and the cubic convolution method. The essence of the nearest point method resampling is to take the gray value of the known pixel point closest to the conjugate position in the original distorted image as the gray value of the output pixel.  Figure 7 shows the gray value interpolation of the output pixel fitting.

The article "Research on the Application of GIS Technology Combined with RBFNN-GA Algorithm in the Delineation of Geological Hazard Prone Areas" was published in 2021. Journal: Comput Intell Neurosci.

Based on the powerful spatial analysis capabilities of GIS, for various geological disaster risk evaluation indicators in a certain area, it is necessary to normalize each indicator to achieve the final comprehensive risk evaluation. In this study, DEM images are downloaded from the geospatial data cloud of the National Academy of Sciences. We use the ArcGIS automatic stitching function to get the DEM map. After SPSS software completes logistic regression analysis, the output digital matrix can also be converted into raster graphics in GIS software, thus solving the problem of mutual import of data in GIS and professional statistical analysis software. In order to unify the coordinates and facilitate the postprocessing, the DEM is converted into general coordinates. According to the distribution of geological hazards, we use Spatial Analyst in ArcGIS density tool to designate a circular area and use a field radius of 1,000 m to analyze the point density of geological hazards. The higher the point density in the area is, the more it reflects, the higher the probability of geological disasters in this area, and the greater the risk of geological disasters is. The data sample set is divided into two parts: the modeling sample set (1,056 data samples) used to build the RBF neural network model and the test sample set (168 data samples). Through calculation, the performance value convergence curve can be drawn when constructing the network. It can be seen that it can converge to the target value after 126 generations.

Figure 8 shows the standard deviation line chart of the RBFNN network band. The data show that the order of the standard deviation of each band is shown in the figure. It is generally believed that there is good agreement between the amount of information of remote sensing images and the image standard deviation; that is, the larger the standard deviation is, the richer the information is. The standard deviation of each band of the image is greater than 3, the largest is 18, the smallest is 3.4, and the average is 9.4, indicating that the information contained in the features is more enriched, and it is feasible to extract land types. The social attribute factors mainly include important engineering facilities such as reservoirs and a small number of oil extraction plants. In some areas, there are a small amount of urban construction and roads, and human engineering activities are relatively weak, so its social attributes are low. The development density of geological disasters and landslides in this area is about 0.3 places/100 km^2^. Among them, there are only 11 unstable slopes in the southern part of the area, which are of low risk. Considering various factors, the geological hazard risk in this area is positioned as medium, which is the risk area in the regional risk assessment.

The article "Research on the Application of GIS Technology Combined with RBFNN-GA Algorithm in the Delineation of Geological Hazard Prone Areas" was published in 2021. Journal: Comput Intell Neurosci.

## 4. Conclusions

This study comprehensively analyzes the main influencing factors that induce regional geological disasters. Based on the theoretical experience and field investigations, the evaluation index system for geological hazards and the regional geological environment quality evaluation index system are established, and the quality characteristics of the regional geological environment are determined. According to the characteristics of the regional geological disaster risk assessment problem, two simple and practical mathematical methods, GIS technology and neural network, are selected to establish the RBFNN-GA algorithm evaluation model, and the final evaluation results are analyzed and compared. Based on ArcGIS as the underlying platform, a spatial graphic database is established. The attribute database is linked by an external database. The evaluation is obtained through secondary development on the basis of the geological spatial database. The analysis module realizes the spatial analysis function. Finally, the fuzzy comprehensive judgment method is used to optimize and select the evaluation index, and the neural network method is used to determine the weight of the evaluation index. A set of scoring standards based on quantitative indicators is formed, and membership functions are used to obtain values; qualitative indicators are evaluated using expert scoring methods to quantify indicators. At the same time, the main geological disasters in the region are the evaluation objects, combined with GIS technology to comprehensively evaluate the susceptibility and zoning of regional urban geological disasters, and the study area is divided into four levels: excellent, good, medium, and poor. The result shows that the evaluation model is reasonable and the system has strong practicability.

## Figures and Tables

**Figure 1:** Hierarchical topology of GIS technology.

The article "Research on the Application of GIS Technology Combined with RBFNN-GA Algorithm in the Delineation of Geological Hazard Prone Areas" was published in 2021. Journal: Comput Intell Neurosci.

**Figure 2:** Fan-shaped diagrams of geological hazard factors.

**Figure 3:** RBFNN-GA algorithm architecture.

**Figure 4:** Quantitative histogram of the susceptibility of geological disasters.

**Figure 5:** RBFNN network evaluation index normalized comparison line chart.

**Figure 6:** TheGIS system geological hazard influence curvature distribution.

**Figure 7:** Gray value interpolation of output pixel fitting.

**Figure 8:** The standard deviation line chart of the RBFNN network band.

**Table 1:** Normalized processing of GIS disaster indicators

Indicator index	Raster calculator	Weight	Curvature (%)
1	Landslides	0.32	13.5
2	Collapses	0.17	22.1
3	Slopes	0.42	31.2
4	Mudslides	0.09	26.4
5	Cracks	0.11	19.6

## Data Availability

The data used to support the findings of this study are available from the corresponding author upon request.
